# The Application of Metagenomic Next-Generation Sequencing in Detection of Pathogen in Bronchoalveolar Lavage Fluid and Sputum Samples of Patients with Pulmonary Infection

**DOI:** 10.1155/2021/7238495

**Published:** 2021-11-08

**Authors:** Wanghui Shi, Shanshan Zhu

**Affiliations:** ^1^Department of Laboratory, The First People's Hospital in Yuhang District, Hangzhou, Zhejiang 311100, China; ^2^Department of Pediatrics, The First People's Hospital in Yuhang District, Hangzhou, Zhejiang 311100, China

## Abstract

**Objective:**

To uncover the application value of metagenomic next-generation sequencing (mNGS) in the detection of pathogen in bronchoalveolar lavage fluid (BALF) and sputum samples.

**Methods:**

Totally, 32 patients with pulmonary infection were included. Pathogens in BALF and sputum samples were tested simultaneously by routine microbial culture and mNGS. Main infected pathogens (bacteria, fungi, and viruses) and their distribution in BALF and sputum samples were analyzed. Moreover, the diagnostic performance of mNGS in paired BALF and sputum samples was assessed.

**Results:**

The pathogen culture results were positive in 9 patients and negative in 13 patients. No statistical differences were recorded on the sensitivity (78.94% vs. 63.15%, *p* = 0.283) and specificity (62.50% vs. 75.00%, *p* = 0.375) of mNGS diagnosis in bacteria and fungus in two types of samples. As shown in mNGS detection, 10 patients' two samples were both positive, 13 patients' two samples were both negative, 7 patients were only positive in BALF samples, and 2 patients' sputum samples were positive. Main viruses mNGS detected were EB virus, human adenovirus 5, herpes simplex virus type 1, and human cytomegalovirus. Kappa consensus analysis indicated that mNGS showed significant consistency in detecting pathogens in two samples, no matter bacteria (*p* < 0.001), fungi (*p* = 0.026), or viruses (*p* = 0.008).

**Conclusion:**

mNGS showed no statistical differences in sensitivity and specificity of pathogen detection in BALF and sputum samples. Under certain conditions, sputum samples might be more suitable for pathogen detection because of invasiveness of BALF samples.

## 1. Introduction

Pulmonary infection is a respiratory tract infection and features high morbidity and mortality globally [1, 2]. Pulmonary infection arises from single pathogen or intertwined pathogens, like bacteria, fungi, viruses, and parasites. Quick and accurate pathogen diagnosis is a challenge despite several detection approaches. Traditional culture is only used for fungal and bacterial tests, which cannot meet clinical requirements due to long time-consuming and low detection rate of positive [3]. Polymerase chain reaction (PCR) and immunological technique possess high sensitivity and specificity while limited testing range of microorganisms [4]. Besides, pathogen identification is confounded by assorted pathogen infection and drug-resistant pathogens [5, 6]. Hence, efficient paths for detection and diagnosis of pulmonary infection pathogens are necessary.

Metagenomic next-generation sequencing (mNGS) is a high-throughput sequencing method with high efficiency and short detection period [7]. The samples used are accessible. Little extracted DNA from samples enables detection and identification of pathogens by this emerging technology. Since its high positive rate in pathogen tests, mNGS has been successfully applied to clinical trials of varying infection diagnosis [8–10]. As reported by Miao et al. [11], mNGS yields higher pathogen identifying sensitivity, especially for viruses, mycobacterium tuberculosis, fungi, and anaerobes. Zhou et al. [12] discovered that mNGS performance is less affected by previous antibiotic exposure than routine culture. In addition, mNGS enhances detection of pulmonary infection pathogens in lung biopsy, with underlying advantages in sensitivity and speed [9]. mNGS is a comprehensive tool that assists in diagnosis of pulmonary infection pathogen [13, 14].

Respiratory tract samples are common sample types for traditional bacteria or fungus culture, including bronchoalveolar lavage fluid (BALF) and sputum, while whether these two samples affect the detection efficiency of mNGS remain disputed. Previous study found that there were differences in the distribution or composition of the strains in sputum and BALF samples, but overall, the detection consistency of sputum and BALF was fairly well [15]. mNGS in pathogen detection of pulmonary infection patient's BALF and sputum samples has been rarely applied and reported. This investigation aimed at assessing and comparing the diagnostic performance of mNGS in detection of pathogens (bacteria, fungi and viruses) in pulmonary infection in BALF and sputum samples.

## 2. Materials and Methods

### 2.1. Object

Pulmonary infection patients (*n* = 32) treated in The First People's Hospital in Yuhang District during March 2019 and April 2020 were retrospectively selected. Specific diagnostic criteria of the infected patients included new or deteriorated focal or diffuse infiltrating lesions according to chest X-ray or computerized tomography (CT) examination. According to hospital pulmonary infection diagnostic criteria issued by American Thoracic Association [16], the included patients met at least the following two criteria: (i) have fever or body temperature ≥ 38°C; (ii) appearance of cough and expectoration accompanied by hypoxia or more serious respiratory symptoms, (iii) with increased leukocytes (blood regular white blood cells ≥ 10.0 × 10^9^/L), and (iv) with clinical signs like pulmonary consolidation and/or moist rale. This investigation has been approved by ethics committee in The First People's Hospital in Yuhang District. Since this study was a retrospective study and the information presented here could not identify specific patients, the informed consent was not used.

### 2.2. Sample Collection and Treatment

Sputum samples were gathered with natural expectoration or disposable sputum suction catheter. BALF samples were gathered by experienced bronchoscope physicians based on standard procedures using fiber bronchoscope 1T-180 (Olympus, Tokyo, Japan). Intervals between sputum and BALF sample collection were less than 24 h. The samples were used for mNGS and routine microbiological detection. The latter included sputum smear and culture, BALF culture, antigen detection, and PCR detection. Since the lack of routine virus detection, no comparison was performed with routine respiratory tract virus detection.

### 2.3. DNA Isolation and Sequencing

DNA was isolated from sputum or BALF samples using TIANamp Micro DNA Kit (DP316, Tiangen Biotech) as manufacturer's specification. DNA was ultrasonicated to obtain fragments 200-500 bp fragments. Thereafter, DNA library was built through end repair, adapter ligation, and PCR amplification. Quality control of DNA library was undertaken with Agilent 2100 Bioanalyzer (Agilent Technologies, Santa Clara, CA, USA). The final library was sequenced on BGISEQ-50 platform (BGI Co., Ltd, Shenzhen, China).

### 2.4. Bioinformatic Analysis

Raw data were pretreated by removal of low-quality reads, residual adapters, and short reads. Reads mapped to human reference genome were deleted by Burrows-Wheeler transform. Afterwards, the residual sequences and microbial genomes database (bacteria, viruses, fungi and parasites) were comparatively analyzed. The databases were downloaded from National Center of Biotechnology Information (NCBI; ftp://ftp.ncbi.nlm.nih.gov/genomes). SOAP web (http://soap.genomics.org.cn/) was used to calculate depth and coverage of every species. The number of unique alignment reads was calculated and standardized to get the number of reads stringently mapped to pathogen species (SDSMRN) and the number of reads stringently mapped to pathogen genus (SDSMRNG). Pathogen detection index of mNGS included specific oligonucleotide read numbers read by the species. Larger read number refers to higher pathogenic bacteria.

### 2.5. Threshold Criteria of mNGS Analysis [7, 9]

Two tables which were categorized based on the sequencing results of each sample referred to bacteria/fungi and virus, respectively. The specifically mapped read number (SMRN) of each microbial taxonomy was normalized to SMRN/20 million (M) of total sequencing reads (SDSMRN, standardized SMRN).

For different microorganisms, the threshold was set as follows: (I) bacteria/mycoplasma/chlamydia: SDSMRNG ≥ 3, (II) DNA virus/fungus: SDSMRN ≥ 3, (III) parasite: SDSMRN ≥ 100, and (IV) mycobacterium tuberculosis complex (MTC): SDSMRNG ≥ 1.

### 2.6. Statistical Analysis

Researched data were analyzed by SPSS 25.0 software (IBM Corp., Armonk, NY, USA). Measurement data were denoted as mean ± standard deviation, and enumeration data were displayed as number and percentage. Chi-square test and consistency test were used to compare the paired samples. For patients with paired culture results, 2 × 2 contingency tables were applied to determine the sensitivity and specificity of mNGS and culture-based diagnosis in sputum and BALF samples. *p* < 0.05 denoted statistically significant.

## 3. Results

### 3.1. Analysis of Patient's Baseline Characteristics

This investigation included a total of 32 pulmonary infection patients (18 males: 56.25%; 14 females: 43.75%), whose average age was 56.35 ± 13.83, and most of whom are 40-60 (59.38%). A total of 17 patients (53.13%) had underlying diseases: 7 type 2 diabetes (21.88%) cases, 5 chronic obstructive pulmonary diseases (15.63%) cases, 2 connective tissue disease cases (6.25%), 2 bronchiectasis cases (6.25%), and 1 case (3.13%) with lung cancer history. Average time from patient's admission to sampling was 3.82 ± 1.00 days (see Table 1).

### 3.2. Analysis of Bacteria and Fungi Culture in BALF and Sputum Samples

Pathogens were detected in bacteria and fungi culture in 19 patient's BALF samples (positive rate: 59.38%). The detection rate of Acinetobacter baumannii (42.86%), Klebsiella pneumoniae (28.57%), and Pseudomonas aeruginosa (21.43%) in bacterial culture ranked the first three in turn. Candida albicans (50.00%) and Candida near smoothing (37.50%) were the main strains detected in fungal culture. Pathogens were detected in bacteria and fungi culture in the 17 patient's corresponding sputum samples (positive rate: 53.13%). The detection rate of Acinetobacter baumannii (30.77%), Pseudomonas aeruginosa (30.77%), and Klebsiella pneumoniae (23.08%) in bacterial culture ranked the first three in turn. Candida albicans (42.86%), Candida near smoothing (28.57%), and Aspergillus flavus (28.57%) were main strains detected in fungal culture. Details were shown in Table 2.

### 3.3. Identification of Pathogenic Species in BALF and Sputum Samples by mNGS

Among the researched 32 pulmonary infection patients, 19 patients' paired results were positive, 8 were negative, and 5 had no paired culture results. mNGS sensitivity in BALF and sputum was 78.94% and 63.15%, respectively, and they had no significant differences (*p* = 0.283). The specificity between mNGS in BALF (5/8 = 62.50%) and sputum (6/8 = 75.00%) samples was not significantly different (*p* = 0.375) (Figure 1).

### 3.4. mNGS Detection of Virus in BALF and Sputum Samples

As provided in Figure 2(a), mNGS results are positive in 10 patient's BALF and sputum samples, negative in 13 patients' BALF and sputum samples, positive in 7 patients' and BALF samples, and positive in 2 patients' sputum samples. Distribution of viruses identified by mNGS in BALF and sputum was shown in Figure 2(b). mNGS-detected viruses in 32 patients were EB virus (EBV), human adenovirus 5, human cytomegalovirus, and herpes simplex virus type 1. EBV was detected in sputum but not in BALF in two patients.

### 3.5. Comparison of Diagnostic Results of mNGS in Pulmonary Infection in BALF and Sputum Samples

Analysis exhibited that bacterial pathogen was found in 17 BALF samples (53.12%) by mNGS assay (Table 3). 16 positive sputum cases (50.00%) were found by the mNGS method. Concordance rate of two samples was 90.63%. Consensus analysis displayed noticeable consensus (*p* < 0.001) and good concordance rate (Kappa = 0.813) between mNGS bacterial detection in two samples. With respect to fungus detection, there were 6 BALF positive samples (18.75%) and 3 positive sputum samples (9.37%), and the concordance rate was 84.38%. Consensus analysis showed notable consensus between mNGS fungus detection of two samples (*p* = 0.026) while concordance rate was low (Kappa = 0.365). Regarding virus detection, there were 17 positive BALF samples (53.13%) and 12 positive sputum samples (37.50%), and concordance rate was 71.88%. Consensus analysis showed noticeable consensus of mNGS detection for virus between two samples (*p* = 0.008), and concordance rate was normal (Kappa = 0.446).

## 4. Discussion

Pulmonary infection is the most prevalent infectious disease with high morbidity and mortality especially for those at old age and with low immunity [2]. Poor efficacy of experiential therapy is mainly attributed to uncertain pathogenic bacteria and compound infection. Quick and accurate detection of infectious pathogens is critical to pulmonary infection patient's treatment and prognosis but is also challenging. Especially in immunocompromised hosts, most bacterium or fungus is potential pathogens for pulmonary infection [7, 17]. mNGS offers unbiased and highly sensitive tests for simultaneously detecting hundreds of pathogens in clinical samples [18]. This investigation performed mNGS and traditional pathogenic detections on 32 pulmonary infection patients' BALF and sputum samples and compared diagnostic performance of mNGS in detection of pathogens (bacteria, fungi, and viruses) in BALF and sputum samples.

Acinetobacter baumannii, Klebsiella pneumoniae, and Pseudomonas aeruginosa were the main strains in the culture of BALF and sputum samples. Candida albicans and Candida near-smoothing were the main strains detected by fungal culture. It can be seen that main positive strains and their distribution in BALF and sputum samples from patients with pulmonary infection were basically the same. The result was similar to a report by Qin et al. [19]. To date, few studies involved comparison of the diagnostic performance of mNGS on pulmonary infection in BALF and sputum samples. The specificity and sensitivity of mNGS in BALF and sputum samples were not noticeably different, which held an agreement with previous research [15].

In the identification analysis of BALF and sputum samples by mNGS, this study found that the detected viruses were mainly EBV, human adenovirus 5, herpes simplex virus type 1, and human cytomegalovirus. EBV was detected in sputum but not in BALF in two patients. In addition, it was also found that the sequence number of human cytomegalovirus detected in BALF mNGS was similar to that in sputum samples, which is consistent with a study finding no statistical difference in the levels of cytomegalovirus DNA between BALF and sputum [20]. Further, it was also compared the diagnostic performance of mNGS in BALF samples and sputum samples in pulmonary infection, and the results showed that the consistent rates of bacteria and fungi detection were 90.63% and 84.38%, respectively. Consensus analysis showed conspicuous consistency in mNGS detection in two samples. The concordance rate of virus detection was 71.88%, and the results of mNGS detection were also significantly consistent. Hence, it was considered that there is no significant difference between the mNGS results in BALF and sputum samples. Under certain conditions, sputum samples might be more suitable for pathogen detection because of invasiveness of BALF.

There are some limitations to this investigation. First, the researched samples were few, which may affect accuracy of evaluation of mNGS performance. Second, mNGS-detected pathogens were not verified by additional molecular assays on a genetic level. Additionally, due to the limitation of time and laboratory conditions, we only conducted mNGs on DNA to detect bacteria, fungi, and DNA viruses, but did not conduct RNA virus detection and further drug sensitivity tests. Lastly, despite advantages of mNGS in pathogen detection, the detection rate for rare strains remains to be improved [21]. In the future, multicenter prospective study with more participators and sample types is needed for incremental evaluation of mNGS application on diagnosis of pulmonary infection.

On the whole, the overall efficiency of mNGS in detection of two samples was similar but the detection efficiency may be affected by pathogen distribution. Furthermore, when the sputum mNGS test results are inconsistent with the clinical symptoms and imaging, especially when invasive pulmonary fungal infection is highly suspected, BALF samples should be taken in time for testing to identify the pathogen species. Drug sensitivity tests of pathogenic bacteria should be carried out in time, so as to provide a reference for rational use of antibiotics and precise treatment in clinical practice.

## Figures and Tables

**Figure 1:** Identification of pathogenic species in BALF and sputum samples by mNGS. (a) Identification of pathogens in BALF and sputum samples in patients with negative culture results. (b) Culture results of 32 patients: 19 positives (blue), 8 negatives (green), and 5 without paired culture results (grey). (c) Identification of pathogens in BALF and sputum samples of patients with positive culture results by mNGS.

**Figure 2:** mNGS detection of viruses in BALF and sputum samples. (a). Results of mNGS virus detection in 32 patients' BALF and sputum samples: 13 patients' mNGS results were allnegative (dark purple); viruses were detected in 19 patients. 10 patients (dark blue) were all positive, 7 patients were BALF positive (light blue), and 2 patients were sputum positive (green). (b) Virus distribution in BALF and sputum samples identified by mNGS. Abbreviations: EBV: Epstein-Barr virus; HAdV: human adenovirus; HCMV: human cytomegalovirus; HSV-1: herpes simplex virus type 1.

**Table 1:** Pulmonary infection patient's baseline characteristics.

Characteristic	Patient, *n* (%)
Sex (%)	
Male	18 (56.25%)
Female	14 (43.75%)
Age (years old)	
≤40	3 (9.37%)
41-60	19 (59.38%)
>60	10 (31.25%)
Underlying disease (%)	
Diabetes	7 (21.87%)
Chronic obstructive pulmonary disease	5 (15.63%)
Connective tissue disease	2 (6.25%)
Bronchiectasis	2 (6.25%)
Lung cancer	1 (3.13%)
Times from admission to sampling (days)	3.82 ± 1.00

**Table 2:** Positive strain constituent in BALF and sputum samples.

BALF sample		Sputum sample	
Pathogenic species	Positive strain constituent, *n* (%)	Pathogenic species	Positive strain constituent, *n* (%)
Bacteria		Bacteria	
Baumanii	6 (42.86%)	Baumanii	4 (30.77%)
Klebsiella pneumoniae	4 (28.57%)	Pseudomonas aeruginosa	4 (30.77%)
Pseudomonas aeruginosa	3 (21.43%)	Klebsiella pneumoniae	3 (23.08%)
Mycobacterium tuberculosis	1 (7.14%)	Mycobacterium tuberculosis	1 (7.69%)
		Escherichia coli	1 (7.69%)
Fungus		Fungus	
Candida albicans	4 (50.00%)	Candida albicans	3 (42.86%)
Nearly smooth Candida	3 (37.50%)	Nearly smooth Candida	2 (28.57%)
Aspergillus flavus	1 (12.50%)	Aspergillus flavus	2 (28.57%)

**Table 3:** Comparison of mNGS detection in pulmonary infection patient's BALF and sputum samples.

Bacteria	Sputum mNGS+	Sputum mNGS-	Fungus	Sputum mNGS+	Sputum mNGS-	Virus	Sputum mNGS+	Sputum mNGS-
BALF mNGS+	15	2	BALF mNGS+	2	4	BALF mNGS+	10	7
BALF mNGS-	1	14	BALF mNGS-	1	25	BALF mNGS-	2	13
Consensus analysis	*p* value	<0.001	Consensus analysis	*p* value	0.026	Consensus analysis	*p* value	0.008
	Kappa	0.813		Kappa	0.365		Kappa	0.446

## Data Availability

The data and materials in the current study are available from the corresponding author on reasonable request.
